The article "Identification of the Upregulation of MRPL13 as a Novel Prognostic Marker Associated with Overall Survival Time and Immunotherapy Response in Breast Cancer" was published in 2021. Journal: Comput Math Methods Med.

# Identification of the Upregulation of MRPL13 as a Novel Prognostic Marker Associated with Overall Survival Time and Immunotherapy Response in Breast Cancer

**DOI:** 10.1155/2021/1498924

**Published:** 2021-11-25

**Authors:** Hongshan Ye, Ning Zhang

**Affiliations:** ^1^Department of Thyroid and Breast Surgery, The 3rd Affiliated Hospital of Shenzhen University, Shenzhen, Guangdong Province, China; ^2^Department of Vascular Surgery, The 3rd Affiliated Hospital of Shenzhen University, Shenzhen, Guangdong Province, China

## Abstract

Mitochondrial ribosomal protein (MRPL) genes have been reported to participate in many cellular processes, such as cell proliferation, apoptosis, and cell cycle. Meanwhile, the occurrence rate of breast cancer (BRCA) in China steadily increased. Exploring the prognostic value of MRPL genes in BRCA could provide novel biomarkers for BRCA. In this study, to identify prognosis-related genes in breast cancer, the *P* value and the hazard ratio (HR) of all genes are analyzed with TCGA database. We revealed higher expression level of CEL, PGK1, WNT3A, USP41, LINC02037, PCMT1, LRP11, MCTS1, TCP1, TMEM31, STK4-AS1, STXBP5, LOC100287036, SLC16A2, MRPL13, DERL1, and TARS was correlated to shorter OS time in BRCA. However, higher expression level of JCHAIN, KLRB1, and TNFRSF14 was correlated to longer OS time in BRCA. The further analysis demonstrated MRPL13 was overexpressed in BRCA. Subtype analysis showed that MRPL13 was overexpressed in luminal, HER2-positive BRCA, and TNBC samples and was highest in TNBC samples. Moreover, we revealed higher expression of MRPL13 was significantly correlated to shorter OS time and higher TMB levels in BRCA. Pan-cancer analysis further revealed the prognostic value of MRPL13 in human cancers. MRPL13 expression was significantly increased in multiple human cancers, such as bladder cancer, colon cancer, liver cancer, and prostate cancer. Pan-cancer TMB and overall survival time showed dysregulation of MRPL13 is significantly related to the OS and TMB levels in various cancers. These results further proved that MRPL13 may be a pan-cancer biomarker for predicting prognosis and the response to immunotherapy.

## 1. Introduction

Breast cancer (BRCA) consisted of endocrine-dependent breast cancer and HER2-positive breast cancer along with triple-negative breast cancer (TNBC) in view of its histological features [1–3]. Recently, the occurrence rate of BRCA is still increasing, and it reached the highest among women [4, 5]. Besides, the occurrence rate of BRCA amid young people has also heightened [4]. Currently, the occurrence rate of BRCA in China steadily increased [6]. The lethality rate of BRCA accounts for about 18% of cancer mortality [1–3, 6, 7]. Present standard treatments against BRCA are mainly composed of surgery, radiotherapy, chemotherapy, hormone therapy, and so on [7]. Targeting receptor tyrosine kinase (RTK) has become an important direction in breast cancer treatment. HER2-targeted treatment therapy significantly improved HER2^+^ BRCA prognosis [8]. Antiestrogen therapy, as the first targeted therapy of human BC, is a treatment of estrogen receptor-positive BC [1, 8, 9]. Therefore, it is urgently needed to uncover early detection biomarkers and explore therapeutic strategies for BRCA.

The article "Identification of the Upregulation of MRPL13 as a Novel Prognostic Marker Associated with Overall Survival Time and Immunotherapy Response in Breast Cancer" was published in 2021. Journal: Comput Math Methods Med.

Mitochondria function importantly in regulating eukaryotic cells' life and death, which mediates the conversion of aerobic energy via the oxidative phosphorylation (OXPHOS) system and conceals and controls cell apoptosis's internal pathway [10–13]. The mitochondrial ribosome comprised a small 28S subunit and a large 39S subunit [10, 12]. Therefore, mitotic ribosomes are the key to regulating cell respiration. There are some studies showing the levels of gene-encoded mitotic ribosomal proteins, mitotic ribosomal assembly factors, and mitochondrial translation factors have changed in several carcinomas [14–16]. Some researches revealed that these changes were probably associated with the occurrence and metastasis of tumor [15]. In recent years, some of the MRPs participated in multiple cellular processes, including cell proliferation, in vitro ribosome cycle regulation, and apoptosis of cells, and MRPL20 expression levels were significantly downregulated in androgen-independent prostate cancer [11, 12, 15]. The levels of MRPL37 and mRNA in different lymphoma tissues were also significantly increased. MRPL33 is necessary for mitochondrial function and is associated with the progression of tumor [11, 15, 17]. Nonetheless, it is not completely understood of the role of mitochondrial ribosomes in BRCA.

Here, we adopted biology tools and experimental validation of the expression of 33 MRPL family members and their possible. These data indicate that MRPL13 and MRPL18 are involved in the progress of BRCA. In order to verify this possibility, we used bioinformatics to study their expression in BRCA and its relationship with prognosis. A prognostic nomogram model based on seven prognostic-related factors is well used to predict the survival rate and provides new insights for the diagnosis and treatment of BRCA.

## 2. Materials and Methods

### 2.1. Survival Analysis

We carried out Kaplan-Meier survival analysis and multivariate Cox regression analysis to evaluate the prognostic value of MRPL genes. According to the median of the expression of each gene, we divided patients into highly expressed group and lowly expressed group. The clinical factors associated with BRCA's prognosis and clinical indicators were separately analyzed by Kaplan-Meier (KM) survival analysis and Cox regression analysis [18]. The Kaplan-Meier plotter is a database used for analyzing the correlation between genes and survival time in 21 cancer types.

The article "Identification of the Upregulation of MRPL13 as a Novel Prognostic Marker Associated with Overall Survival Time and Immunotherapy Response in Breast Cancer" was published in 2021. Journal: Comput Math Methods Med.

### 2.2. Data Preparation

We analyzed mRNA expression data from The Cancer Genome Atlas (TCGA, http://tcga-data.nci.nih.gov/tcga) [19].

### 2.3. Bioinformatics Analysis

To determine the distribution of MRPL genes in BRCA tumors and normal tissues, we conducted the gene expression profile interaction analysis (GEPIA) (http://gepia.cancer-pku.cn/) to obtain a box diagram of MRPL genes [20]. We carried out annotation, visualization and integrated discovery database (DAVID) v.6.8 [21], and BINGO (https://www.psb.ugent.be/cbd/papers/BINGO/Home) [22] to analyze enriched functions.

### 2.4. MRPL-Related Gene Analysis in BRCA

We applied Pearson correlation coefficient analysis [23] to evaluate the MRPL-associated genes in BRCA. The correlation coefficient *R* ≥ 0.4 or *R* ≤ −0.4 is considered highly correlated. *P* value ≤ 0.01 means significantly statistical difference.

### 2.5. Clinical Significance of MRPL Genes in BRCA

In view of the median of the expression of each gene, we divided patients into highly expressed group and lowly expressed group. The Kaplan-Meier estimator is used to determine the correlation of gene expression with patients' overall survival rate (OS). We adjusted the multivariate Cox proportional hazards regression model in the light of tumor stage.

### 2.6. Nomogram for Predicting BRCA's Prognosis

We constructed nomogram to predict BRCA's prognosis and risk scores. This model contained all MRPL genes and clinical details. We calculated the points corresponding to each parameter and then evaluated the correlation of obtained points with the risk. We predicted 1-year, 5-year, and 10-year prognostic status [24, 25].

### 2.7. Statistical Analysis

We evaluated the differences in survival rates existing in the two groups according to hazard ratios (HRs) and 95% confidence intervals (CIs). SPASS version 25.0 (IBM, USA) and Graphpad version 7.0 (LaJolla, USA) were applied for statistical analysis and mapping. *P* < 0.05 means greatly statistical differences between the two groups.

## 3. Results

### 3.1. Identification of Prognosis-Related Genes in Breast Cancer

In order to identify prognosis-related genes in breast cancer, the *P* value and the hazard ratio (HR) of all genes are analyzed with TCGA database. The top 20 significantly genes related to the prognosis of breast cancer are listed in Figure 1. Among them, higher expression level of CEL, PGK1, WNT3A, USP41, LINC02037, PCMT1, LRP11, MCTS1, TCP1, TMEM31, STK4-AS1, STXBP5, LOC100287036, SLC16A2, MRPL13, DERL1, and TARS was correlated to shorter OS time in BRCA (Figure 1). However, higher expression level of JCHAIN, KLRB1, and TNFRSF14 was correlated to longer OS time in BRCA (Figure 1). Interestingly, we observed several lncRNAs were significantly related to prognosis in breast cancer, such as LINC02037 and STK4-AS1. Among these genes, we focused on MRPL13, whose function in BRCA remained largely unclear.

The article "Identification of the Upregulation of MRPL13 as a Novel Prognostic Marker Associated with Overall Survival Time and Immunotherapy Response in Breast Cancer" was published in 2021. Journal: Comput Math Methods Med.

### 3.2. The Expression and Protein Levels of MRPL13 Were Upregulated in BRCA

In order to further confirm the upregulation of MRPL13 in BRCA, we used the UALCAN database to evaluate MRPL13 gene and protein levels in BRCA.  Figure 2 illustrates that MRPL13 RNA and protein levels in BRCA are significantly higher than normal samples (Figures 3(a) and 3(b)). Additionally, subtype analysis showed that MRPL13 was overexpressed in luminal, HER2-positive BRCA, and TNBC samples and was higher in TNBC samples than the two former samples (Figures 3(c) and 3(d)).

### 3.3. Constructing and Evaluating the Nomogram for MRPL13

We also analyzed univariate and multivariate Cox proportional hazards and found that three general variables (age, gender, and TNM staging) and two genes (MRPL13 and MRPL18) presented great difference existing in the nonrelapsed and the relapsed groups (Figures 2(a) and 2(b)). We constructed a nomogram to calculate the recurrence risk of each patient through the points related to MRPL13 and MRPL18 on the basis of the multivariate Cox proportional hazard analysis. The total score is 0-160 points, and the variables are calculated and combined (Figure 2(c)). After comparison with the expected model in the whole cohorts, we concluded that the calibration plots for 1-year, 3-year, and 5-year OS rates presented well prediction (Figure 2(d)).

### 3.4. Overexpression of MRPL13 Was Correlated to Shorter OS in BRCA

Next, we conducted further analysis on MRPL13 in BRCA. According to the median expression of MRPL13 in BRCA, we separated BRCA patients into MRPL13 highly expressed group and MRPL13 lowly expressed group.  Figure 4(a) shows that high expression levels are associated with more deaths. KM survival curves showed that BRCA patients with highly expressed MRPL13 exhibited shorter OS than those with lowly expressed MRPL13 (Figure 4(b)). The AUC values of 1-year, 3-year, 5-year, 10-year, and 15-year survival rate prediction features are 0.605, 0.605, 0.595, 0.586, and 0.528, respectively (Figure 4(c)).

### 3.5. The Confirmation of Correlation between MRPL13 Expression and Prognosis

Next, we use the KM database to confirm the association of MRPL13 expression with prognosis. Our results show that BRCA patients with highly expressed MRPL13 displayed shorter OS, RFS, PPS, and DMF time (Figures 5(a)–5(d)). Further, subtype analysis showed that luminal A, luminal B, of HER2-positive, and TNBC patients with high levels of MRPL13 expression had shorter RFS time (Figures 5(e)–5(h)).

The article "Identification of the Upregulation of MRPL13 as a Novel Prognostic Marker Associated with Overall Survival Time and Immunotherapy Response in Breast Cancer" was published in 2021. Journal: Comput Math Methods Med.

### 3.6. Overexpression of MRPL13 Was Correlated to Higher TMB Levels in BRCA

Tumor mutational burden (TMB) is a promising biomarker for predicting tumor immunotherapy response. Here, we assessed the relationship of MRPL13 expression with TMB levels. Our results show that higher expression of MRPL13 was correlated to higher TMB levels in BRCA, luminal A BRCA, luminal B BRCA, and HER2-enriched BRCA patients (Figures 6(a)–6(d)). Nevertheless, there is no greatly significant correlation of MRPL13 with TMB level in TNBC patients (Figure 6(e)).

### 3.7. Expression Levels of MRPL13 Were Correlated to OS Time and TMB Levels in Pan-Cancer

In addition, three different databases based on TCGA cohort were used to evaluate the expression of MRPL13 mRNA in 33 cancer types. TIMER database results have shown that MRPL13 expression in certain cancers were significantly increased, including the BLCA, the BRCA, CESC, CHOL, COAD, ESCA, GBM, HNSCs, LIHC, LUAD, LUSC, PRAD, Read, the STAD, and UCEC (Figures 7(a)–7(d)). However, MRPL13 expression was reduced in KICH, KIRC, and PCPG (Figures 7(a)–7(d)).

We also analyzed the association of MRPL13 expression in pan-carcinoma MRPL13 expression with TMB and OS. Our results show that the dysregulation of MRPL13 is significantly related to the OS of ACC, BRCA, KICH, LAML, LGG, LIHC, LUAD, PAAD, SARC, and UVM (Figure 8(a)).

In addition, we also analyzed the correlation of MRPL13 expression with TMB in human cancer. Our results show that MRPL13 expression exhibited a significantly positive correlation with TMB levels of DLBC, STAD, PAAD, BRCA, LUAD, UCS, SARC, LGG, PRAD, and LUSC, while presented a significantly negative correlation with the TMB levels of thymus, UVM. These results further prove that MRPL13 may be a pan-cancer biomarker for predicting response to immunotherapy (Figure 8(b)).

## 4. Discussion

In this study, we identified prognosis-related genes in breast cancer. Interestingly, we observed several lncRNAs were significantly related to prognosis in breast cancer, such as LINC02037 and STK4-AS1. Previous studies had revealed these lncRNAs have a crucial role in human cancers. For example, Li et al. reported LINC02037 was differently expressed in breast cancer and could predict prognosis of breast cancer patients. In recent years, some MRPs have been reported to participate in many cellular processes, such as cell proliferation, apoptosis, and cell cycle [10, 14–16]. The growing researches have reported that the abnormally expressed MRPs exhibited a relationship to human tumors' occurrence and development [15, 16]. For example, MRPL15 is a new prognostic indicator and therapeutic target for epithelial ovarian cancer [26]. MRPS12 is a potential oncogene of ovarian cancer [27], while MRPL27 displays an adverse effect on the overall survival rate and disease-free survival rate of cholangiocarcinoma patients [28]. MRPL42 is activated by YY1 to promote the progression of lung adenocarcinoma [29]. MRPL42 gene knockout inhibits the proliferation of glioma cells by inducing cell cycle arrest and apoptosis [30]. Here, we analyzed TCGA data and performed bioinformatics to reveal potential prognostic value of MRPL genes in BRCA. The results indicate significant difference exists in MRPL family gene (including MRPL1, MRPL13, and MRPL18) expression between BRCA tissues and normal tissues. Survival analysis showed that the overexpression of MRPL1, MRPL13, and MRPL18 was associated with a shorter OS time in BRCA.

The article "Identification of the Upregulation of MRPL13 as a Novel Prognostic Marker Associated with Overall Survival Time and Immunotherapy Response in Breast Cancer" was published in 2021. Journal: Comput Math Methods Med.

Mitochondrial ribosomal protein L13 (MRPL13) is located on chromosome 6 and encodes the 39S large subunit of mitochondrial ribosomes [31, 32]. MRPL13 is a predictive biomarker of BRCA and exhibits a relationship to the immune infiltration of BRCA. MRPL13 mediated the promotion of BRCA cells' proliferation, migration, and EMT process through PI3K-AKT-mTOR pathway [32]. siRNA-mediated knockout of MRPL13 reduces the expression of mitochondrial protein in SNU387 cells, reduces oxygen consumption, and increases CLN1-mediated tumor cell invasiveness [33–35]. Nevertheless, it is still elusive towards MRPL13's role in BRCA. Here, we tested MRPL13 expression in normal tissues, various cell lines, and pan-cancer. Our results show that the expression of MRPL13 in BRCA is higher than that in normal people. Subtype analysis shows that MRPL13 is overexpressed in luminal, HER2-positive, and TNBC samples and is higher in TNBC samples than the former samples. Moreover, high expression of MRPL13 is related to poor prognosis of BRCA. These results suggest MRPL13 is a potential marker for BRCA prognosis.

Traditionally, BRCA is considered as a low immunogenic disease (so-called “cold” tumor) because of its low mutation burden, low number of tumor infiltrating lymphocytes (TIL), and low expression of programmed cell death protein/ligand (PD-1/L1) [36–38]. Preclinical and clinical trials have shown that immunotherapy is an emerging method for BRCA treatment. Recently, nivolumab (anti-PD-1mAb) and ipilimumab (anti-CTLA-4-mAb) have been applied in phase I/II trial of TNBC treatment and achieved well clinical efficacy [36–40]. The use of several immunotherapy agents as a single treatment for metastatic triple-negative BRCA has also shown a moderate but long-lasting response rate and tolerable safety [40, 41]. However, the clinical application of immunotherapy is limited because the efficacy of immunotherapy agents is still very low [41, 42]. Therefore, there is an urgent need to use new biomarkers to predict the response of BRCA to immunotherapy. TMB is related to a variety of tumor immunogenicity indicators and has been proven to have clinical application value in carcinomas [43]. Higher TMB value was observed in TNBC than other subtypes of BRCA. Recently, some studies show that TNBC cases with high TMB perhaps benefit from immune checkpoint blockade along with chemotherapy or immune checkpoint blockade alone [40–44]. As a potential toolset, TMB could be utilized as a helper for TNBC patients [44]. Currently, we firstly demonstrated that increase level of MRPL13 is significantly related to the increase of TMB value in TNBC. In addition, we also analyzed MRPL13 with TMB relation human cancers, and the results show that MRPL13 and DLBC, STAD, PAAD, BRCA, LUAD, UCS, SARC, LGG, PRAD, and LUSC in TMB were significantly positively correlated with elevated levels. And it is negatively correlated with the increase of TMB levels in thymus, UVM. These results further prove that MRPL13 may be a pan-cancer biomarker for predicting response to immunotherapy.

The article "Identification of the Upregulation of MRPL13 as a Novel Prognostic Marker Associated with Overall Survival Time and Immunotherapy Response in Breast Cancer" was published in 2021. Journal: Comput Math Methods Med.

Finally, this study has some limitations. First of all, this research is based on bioinformatics analysis, and its potential biological mechanism needs to be further studied. Second, we would conduct more researches to investigate the protein expression level of MRPL13 and its role in the pathogenesis and progression of BRCA. We firstly revealed the potential association of MRPL gene expression with BRCA tumor immune escape and fully explored the role of MRPL gene in BRCA patients. Our findings would offer some certain reference value for the research and clinical treatment of BRCA.

In short, the high expression of MRPL3 predicts a poor prognosis of BRCA, so it may be a potential biomarker of the disease. These genes can regulate BRCA tumor-related signaling pathways and inhibit the immune infiltration of BRCA tumors. Further prospective studies are needed to verify these molecular mechanisms.

## Figures and Tables

**Figure 1:** Identification of prognosis-related genes in breast cancer. The top 20 significantly genes related to the prognosis of breast cancer are listed in Figure 1.

The article "Identification of the Upregulation of MRPL13 as a Novel Prognostic Marker Associated with Overall Survival Time and Immunotherapy Response in Breast Cancer" was published in 2021. Journal: Comput Math Methods Med.

**Figure 2:** Constructing and evaluating the nomogram for MRPL13. (a) Univariate analysis and (b) multivariate analysis of the correlation between MRPL13 and overall survival in BRCA. (c) The nomogram is constructed for MRPL13 in BRCA. (d) Calibration curves of the nomogram for the prediction of survival rates at 1, 3, and 5 years.

**Figure 3:** MRPL13 is overexpressed in BRCA. (a) The RNA levels of MRPL13 are overexpressed in BRCA compared to normal samples. (b) The RNA levels of MRPL13 are different among normal samples, luminal BRCA, HER2-positive BRCA, and TNBC. (c) The protein levels of MRPL13 are overexpressed in BRCA compared to normal samples. (d) The protein levels of MRPL13 are different among normal samples, luminal BRCA, HER2-positive BRCA, and TNBC. The *P* value was calculated by the unpaired two-tailed Student's *t*-test. ^∗^*P* < 0.05, ^∗∗^*P* < 0.01, and ^∗∗∗^*P* < 0.001.

**Figure 4:** Higher expression level of MRPL13 was correlated to shorter OS in BRCA. (a) From top to bottom are the expression values of MRPL13, patients' survival status distribution, and the heatmap of MRPL13 expression in the low and high groups. (b) Higher expression level of MRPL13 was correlated to shorter OS in BRCA. (c) AUC analysis of MRPL13 in BRCA.

**Figure 5:** The confirmation of correlation between MRPL13 expression and prognosis. (a–d) highly expressed MRPL13 displayed shorter (a) RFS, (b) PPS, (c) OS, and (d) DMFS time. (e–h) Subtype analysis showed that (e) luminal A, (g) luminal B, (h) HER2-positive, and (f) TNBC patients with high levels of MRPL13 expression had shorter RFS time.

**Figure 6:** Higher expression of MRPL13 was correlated to higher TMB levels in BRCA. (a–e) Our results show expression of MRPL13 was correlated to TMB levels in BRCA, luminal A BRCA, luminal B BRCA, HER2-enriched BRCA, and TNBC patients.

**Figure 7:** Pan-cancer analysis showed MRPL13 was upregulated in BRCA.

**Figure 8:** Pan-cancer analysis showed MRPL13 was correlated to OS and TMB levels in human cancers. (a) Pan-cancer analysis showed MRPL13 was correlated to OS in human cancers. (b) Pan-cancer analysis showed MRPL13 was correlated to TMB levels in human cancers.

## Data Availability

The data used in the current study are available from the GEO (https://www.ncbi.nlm.nih.gov) and TCGA (https://portal.gdc.cancer.gov/).
